RETRACTED

# Degradation of long non-coding RNA-CIR decelerates proliferation, invasion and migration, but promotes apoptosis of osteosarcoma cells

**DOI:** 10.1186/s12935-019-1076-7

**Published:** 2019-12-23

**Authors:** Shiwei Liu, Jingchao Li, Liang Kang, Yueyang Tian, Yuan Xue

**Affiliations:** 1 Department of Orthopaedics, Tianjin Medical University General Hospital, 154 Anshan Road, Heping District, Tianjin, 300052 China; 2 Tianjin Key Laboratory of Spine and Spinal Cord, Tianjin Medical University General Hospital, 154 Anshan Road, Heping District, Tianjin, 300052 China

**Keywords:** Osteosarcoma, Long non-coding RNA cartilage injury-related, Proliferation, Invasion, Migration, Apoptosis

## Abstract

**Background:**

Over the years, long non-coding RNAs (lncRNAs) have been clarified in malignancies, this research was focused on the role of lncRNA cartilage injury-related (lncRNA-CIR) in osteosarcoma cells.

**Methods:**

LncRNA-CIR expression in osteosarcoma tissues and cells, and adjacent normal tissues and normal osteoblasts was determined, then the relations between lncRNA-CIR expression and the clinicopathological features, and between lncRNA-CIR expression and the prognosis of osteosarcoma patients were analyzed. Moreover, the MG63 and 143B cells were treated with silenced or overexpressed lncRNA-CIR, and then the proliferation, invasion, migration and apoptosis of the cells were evaluated by gain- and loss-of-function approaches. The tumor growth, and proliferation and apoptosis of osteosarcoma cells in vivo were observed by subcutaneous tumorigenesis in nude mice.

**Results:**

We have found that lncRNA-CIR was up-regulated in osteosarcoma tissues and cells, which was respectively relative to adjacent normal tissues and normal osteoblasts. The expression of lncRNA-CIR was evidently correlated with disease stages, distant metastasis and differentiation of osteosarcoma patients, and the high expression of lncRNA-CIR indicated a poor prognosis. Furthermore, the reduction of lncRNA-CIR could restrict proliferation, invasion and migration, but promote apoptosis of osteosarcoma cells in vitro. Meanwhile, inhibited lncRNA-CIR also restrained tumor growth and osteosarcoma cell proliferation, whereas accelerated apoptosis of osteosarcoma cells in vivo.

**Conclusion:**

We have found in this study that the inhibited lncRNA-CIR could decelerate proliferation, invasion and migration, but accelerate apoptosis of osteosarcoma cells, which may provide a novel target for osteosarcoma treatment.

## Background

Osteosarcoma is the most frequent primary malignant bone tumor in children and adolescents [1]. The commonest location of osteosarcoma is the metaphysis of long bones with the most common site being the distal femur, which is followed by the proximal tibia and humerus. Although common in the long bones of the extremities, osteosarcoma can be diagnosed in any bone [2]. The incidence of osteosarcoma is three cases per million. The 5-year survival rate of patients with localized osteosarcoma is 80%, while that of patients with metastatic osteosarcoma is 15–30% [3]. The pathogenesis of osteosarcoma is comprised of genetic and environmental factors. At present, the therapy of osteosarcoma involves surgical resection combined with radiotherapy and chemotherapy, which could contribute to prolonged survival. However, high incidence of recurrence and metastasis causes a poor prognosis of osteosarcoma [4]. Therefore, confirming the causative factors is of great significance to promote the treatment and heighten the overall survival rate of patients with osteosarcoma.

RETRACTED

According to the length of the transcript, non-coding RNAs can be separated into small (< 200 nucleotides in length) and long non-coding RNAs (lncRNAs, > 200 nucleotides in length) [5]. Emerging evidence indicates that particular lncRNAs are important for control of gene expression [6]. As previously reported, several particular lncRNAs, such as lncRNA OIP5-AS1 [7] and lncRNA HOXD-AS1 [8] were implicated in osteosarcoma progression. In spite of some progresses so far, the functional mechanisms of lncRNAs in human diseases remain to be elucidated. The aberrant expression of lncRNAs is critically involved in a variety of diseases, particularly cancer. Previously, Liu et al. [9] identified that lncRNA cartilage injury-related (lncRNA-CIR) may increase the degradation of chondrocyte extracellular matrix in osteoarthritis (OA). A study by Li et al. [10] indicated that lncRNA-CIR could promote chondrocyte extracellular matrix degradation in OA by acting as a sponge for microRNA-27b. Wang et al. [11] have found that lncRNA-CIR was able to promote articular cartilage degeneration in OA by regulating autophagy. Meanwhile, lncRNA-CIR has been proved to be up-regulated in bladder cancer tissues and cell lines [12]. Based on these data, we speculate that lncRNA-CIR may be associated with bone diseases and overexpressed in cancer tissues. However, the impact of lncRNA-CIR on the progression of osteosarcoma has not been investigated yet. To further unravel the effect of lncRNA-CIR on human diseases, we conducted this research to explore the role of lncRNA-CIR in osteosarcoma development, and we speculate that the function of lncRNA-CIR may be related to the malignant phenotypes of osteosarcoma cells in vitro and osteosarcoma tumor growth in vivo.

## Materials and methods

### Ethics statement

Written informed consents were acquired from all patients before this study. The protocol of this study was confirmed by the Ethic Committee of Tianjin Medical University General Hospital. Animal experiments were strictly in accordance with the Guide to the Management and Use of Laboratory Animals issued by the National Institutes of Health. The protocol of animal experiments was approved by the Institutional Animal Care and Use Committee of Tianjin Medical University General Hospital.

RETRACTED

### Study subjects

Tumor and adjacent normal tissue samples were harvested from 54 patients with osteosarcoma that have accepted resection in Tianjin Medical University General Hospital from January 2012 to December 2014. All the tumor samples have been diagnosed as osteosarcoma and were preserved in liquid nitrogen. Patients that have accepted intervening measures such as chemotherapy were excluded. The histological classification was in line with the standards that proposed by Dahlin et al. [13] and the tumor staging was in accordance with that proposed by Enneking et al. [14].

### Cell culture

Human osteosarcoma cell lines MG63 and 143B, and human osteoblasts hFOB1.19 were cultured by Dulbecco’s modified Eagle medium (DMEM) containing 10% fetal bovine serum (FBS) and 1% penicillin–streptomycin (P/S), and the human osteosarcoma cell lines U2OS and SAOS2 were cultured by McCoy’s 5A medium containing 20% FBS and 1% P/S. All the cells were obtained from American Type Culture Collection (ATCC, VA, USA), and the DMEM, McCoy’s 5A, FBS and P/S were acquired from Gibco Laboratories (Grand Island, USA).

The cells were seeded in T25 culture flasks, which were appended with medium containing 10% FBS, and then incubated at 37 °C with 5% CO_2_, the medium was changed every 2–3 days. Cells in the logarithmic growth phase were detached by trypsin and passaged at 1:4 when the cell confluence reached 70–80%. Cells in the logarithmic growth phase were selected for the subsequent experiments.

### Cell grouping and transfection

MG63 and 143B cells were seeded onto 12-well plates with each well supplemented with P/S-free complete medium, and then the cells were transiently transfected with short hairpin RNA-negative control (sh-NC), sh-CIR, overexpressed (oe)-NC and oe-CIR based on the instructions of Lipofectamine™ 2000 reagent (Invitrogen Inc., Carlsbad, CA, USA). After 24-h incubation, the medium was replaced by DMEM containing 10% FBS and the cells were incubated for 48 h for subsequent experiments. The control group (cells were transfected without any sequence) was also set. The sh-NC, sh-CIR, oe-NC and oe-CIR were all purchased from GenePharma Co., Ltd. (Jiangsu, China).

RETRACTED

### Reverse transcription quantitative polymerase chain reaction (RT-qPCR)

The total RNA in tissues and cells was extracted by Trizol method (TaKaRa Biotechnology Co., Ltd., Liaoning China) and the purity and concentration of the RNA were determined. Next, the RNA was reversely transcripted into cDNA by PrimeScript RT kits (TaKaRa). The PCR was conducted by ABI PRISM^®^ 7300 system (Applied Biosystems, Inc., CA, USA) and the data were analyzed by 2^−∆∆Ct^ method [15]. Glyceraldehyde phosphate dehydrogenase (GAPDH) was taken as the internal reference, the primers of lncRNA‐CIR and GAPDH (Table 1) were designed by Sangon Biotechnology Co., Ltd. (Shanghai, China).

**Table 1:** Primer sequence

Gene	Primer sequence (5′-3′)
LncRNA‐CIR	Forward: 5′-ACACTTGCAAGCCTGGGTAG-3′
	Reverse: 5′-CCATTTTCCTGTTGGTGCGG-3′
GAPDH	Forward: 5′-TCTCCCTCACAATTTCCATCCC-3′
	Reverse: 5′-TTTTTGTGGGTGCAGCGAAC-3′

*lncRNA-CIR* long non-coding RNA cartilage injury-related, *GAPDH* glyceraldehyde phosphate dehydrogenase

### Western blot analysis

The total protein in tissues and cells was extracted with the concentration assessed. The 10% sodium dodecyl sulfate separation gel and spacer gel were prepared, and the samples were mixed with loading buffer and boiled at 100 °C for 5 min. After conducted with ice bath, centrifugation and electrophoretic separation, the proteins were transferred onto the polyvinylidene fluoride membranes, which were blocked with 5% skim milk powder at 4 °C overnight. Next, the membranes were added with primary antibodies Bcl-2, Bax (both 1:500 and from Proteintech Group Inc., Chicago, USA), proliferating cell nuclear antigen (PCNA), Ki-67, GAPDH (all 1:1000 and from Santa Cruz Biotechnology, Inc, Santa Cruz, CA, USA), matrix metalloproteinase (MMP)2 (1:500) and MMP9 (1:1000, both from Abcam Inc., Cambridge, MA, USA) for overnight incubation. Subsequently, the membranes were appended with secondary antibody horseradish peroxidase-conjugated immunoglobulin G (1:1000, Cell Signaling Technologies, Beverly, MA, USA) and incubated at 37 °C for 1 h, and then soaked in enhanced chemiluminescent reaction solution (Thermo Fisher Scientific Inc., Waltham, MA, USA) for 1 min. With the liquid removed, the membranes were covered by food wrap, and then exposed in dark, developed and fixed. GAPDH was taken as the loading control. The protein bands were analyzed by ImageJ2x software (National Institutes of Health (NIH), Bethesda, Maryland, USA).

### Cell counting kit (CCK-8) assay

MG63 and 143B cells were detached by 0.25% trypsin and the survival cells were counted by trypan blue staining. Cells that have been diluted by DMEM containing FBS were seeded onto 96-well plates at 2000 cells/well and cultured at 37 °C with 5% CO_2_. Each well was supplemented with 10 μL CCK-8 solution when the cells were incubated for 24 h, 48 h and 72 h, respectively. After the 96-well plates incubated for 3 h, the optical density (OD) value at 450 nm was measured by a microplate reader.

RETRACTED

### Colony formation assay

The cells were detached by 0.25% trypsin and the survival cells were counted by trypan blue staining. Cells that have been diluted by DMEM containing FBS were seeded into 6-cm dishes at 1000 cells/10 mL and cultured at 37 °C with 5% CO_2_ for 12–15 days with the medium discarded. After rinsed by phosphate buffered saline (PBS) twice, the cells were fixed by 10 mL 4% paraformaldehyde for 20 min, stained by crystal violet dye for 30 min and observed under a microplate. The colonies were counted.

### 5-Ethynyl-2′-deoxyuridine (EdU) assay

The cells were seeded into 96-well plates and incubated at 37 °C for 24 h, then fixed by 4% formalin for 30 min and permeabilized by 0.5% Triton X-100 for 10 min. Afterwards, the cells were stained in line with the directions of EdU kits (RiboBio Co., Ltd., Guangdong, China): the cells were stained by EdU solution (red) for 1 h and counterstained by Hoechst33342 (blue) for 30 min, then observed under a laser scanning confocal microscope (Nikon Corporation, Tokyo, Japan).

### Terminal deoxynucleotidyl transferase-mediated dUTP nick end-labeling (TUNEL) staining

The cells were seeded into 96-well plates and incubated at 37 °C for 24 h, then added with 100 μL stationary liquid. Next, the cells were stained in accordance with the manufacture’ instructions of TUNEL kits (Maibio Co., Ltd., Shanghai, China): cells were added with 50 μL 4′,6-diamidino-2-phenylindole 2 hci for 10 min and sealed by 120 μL anti-fluorescence quenching reagent, then observed and photographed under a fluorescence microscope (Olympus Optical Co., Ltd, Tokyo, Japan).

### Flow cytometry

Cells in each group were centrifuged at 4 °C and 1000 rpm for 5 min, rinsed by 4 °C pre-cooled PBS twice, centrifuged at 1000 rpm for 5 min with the supernatant removed, and resuspended by 250 μL binding buffer solution. The cell concentration was adjusted to 1 × 10^6^ cells/mL. The cells suspension (100 μL) was added with 5 μL Annexin V-activated protein C (APC) and 5 μL propidium iodide (PI) solution in a 5 mL flow tube, and then incubated without light exposure for 15 min. After the tube supplemented with 400 μL PBS, the results were analyzed by a flow cytometer and a computer.

### Scratch test

Cells were seeded into 6-well plates at 5 × 10^5^ cells/well and covered the plates on the 2nd day; three parallel marks were scratched along the margin of a disinfected ruler in each well by a 200 μL pipette tip. With the supernatant removed, the cells were added with serum-free medium and photographed under a microscope after 24 h. The migration rate of cells in each group was calculated by Image J software (NIH, Bethesda, Maryland, USA).

RETRACTED

### Transwell assay

Matrigel (Nobleryder Technology Co., Ltd., Beijing, China) that have been preserved at − 20 °C were dissolved and mixed with DMEM at 1:8, which was then added into the Transwell chambers (40 μL/chamber), and the chambers were incubated at 37 °C for 4 h. Cells were detached and resuspended to 3 × 10^5^ cells/mL with serum-free medium, and the resuspended cells (150 μL) were supplemented into the apical chambers. The basolateral chambers were appended with 600 μL DMEM containing 10% FBS and incubated for 24 h (3 duplicates were set in each group). Subsequently, the cells were fixed by formalin for 0.5 h, stained by crystal violet dye and photographed under a microscope. The transmembrane cells were counted.

### Experimental animals

An amount of 30 BALB/c nude mice (aging 4 week) that purchased from the Laboratory Animal Center of Chongqing National Biological Industrial Base (Chongqing, China) were fed with sterilized food in specific pathogen-free animal rooms (temperature at 26–28 °C, humidity at 40–60%, 12 h day/night cycle and without particular pathogen).

### Subcutaneous tumorigenesis in nude mice

MG63 and 143B cells were detached by 0.25% trypsin and centrifuged, and the concentration of the cells suspension was modulated to 1 × 10^6^ cells/200 μL, then 200 μL cell suspension was injected into the right lower lateral subcutaneous tissue of the nude mice. The animal grouping was similar to the cellular experiment: the control group, the sh-NC group, the sh-CIR group, the oe-NC group and the oe-CIR group (5 nude mice in each group). The volume of the xenografts was measured and recorded every 7 days and the mice were euthanized on the 6th week with the tumors separated and weighed. The tumor volume (mm^3^) = 0.5 × the longest diameter × the shortest diameter^2^. The harvested xenografts were then conducted with apoptosis detection and immunohistochemical staining (Ki-67 protein expression determination).

Apoptosis detection: the steps were in line with instructions of TUNEL kits (Solabio Life Sciences Co., Ltd, Beijing, China) and the results were observed under a light microscope.

Proliferation of osteosarcoma cells: immunohistochemical staining was employed to measure the protein expression of Ki-67 in osteosarcoma tissues. The rabbit anti-human Ki-67 monoclonal antibody (1:100) was acquired from Dako Inc. (Glostrup, Denmark), and the secondary antibody (1:200) was labeled by biotin. The paraffin tissues were cut into 4-μm sections, which were then conducted with streptavidin-peroxidase assay (Biolab technology Co., Ltd., Beijing, China): the sections were soaked in 0.01 mmol/L citrate buffer solution for antigen retrieval, developed by diaminobenzidine and counterstained by hematoxylin, then dehydrated, permeabilized and sealed. The results were observed under a light microscope. Ki-67 protein expressed in nuclei and the nuclei that stained into brownish yellow or brown indicated the Ki-67 positive expression.

RETRACTED

### Statistical analysis

All data analyses were conducted using SPSS 22.0 software (IBM Corp. Armonk, NY, USA). The measurement data conforming to the normal distribution were expressed as mean ± standard deviation. The unpaired t-test was performed for comparisons between two groups and one-way analysis of variance (ANOVA) was used for comparisons among multiple groups, and Tukey’s post hoc test was used for pairwise comparisons after one-way ANOVA. Classified variable was analyzed by Fisher’s exact test, the survival of patients was analyzed by Kaplan–Meier method, and the difference of the curves was compared by Log-rank test. Cox’s proportional hazards regression was employed for multivariate analysis of prognostic factors. *P* value < 0.05 was indicative of statistically significant difference.

## Results

### LncRNA-CIR is up-regulated in osteosarcoma tissues and cells, and the highly-expressed lncRNA-CIR indicates a poor prognosis of osteosarcoma patients

To determine the expression of lncRNA-CIR in osteosarcoma, RT-qPCR was used to measure lncRNA-CIR expression in osteosarcoma tissues and cell lines. As assessed by RT-qPCR (Fig. 1a, b), lncRNA-CIR expression in 54 osteosarcoma tissues was higher than that in the adjacent normal tissues; lncRNA-CIR expression in human osteosarcoma cells MG63, 143B, U2OS and SAOS2 was higher than that in normal osteoblast hFOB1.19, and there existed an apparent difference in lncRNA-CIR expression between MG63 and 143B cells (all *P *< 0.05). Thus, we chose MG63 and 143B cells for the subsequent experiments.

**Fig. 1:** LncRNA-CIR is up-regulated in osteosarcoma tissues and cells, and the highly-expressed lncRNA-CIR indicates a poor prognosis of osteosarcoma patients. **a** LncRNA-CIR expression in osteosarcoma tissues and adjacent normal tissues; **b** LncRNA-CIR expression in hFOB1.19, MG63, 143B, U2OS and SAOS2 cells; **c** Relation between lncRNA-CIR expression and prognosis of osteosarcoma patients; **d** LncRNA-CIR expression in MG63 cells of each group; **e** LncRNA-CIR expression in 143B cells of each group; the normal group and the tumor group: n = 54, hFOB1.19, MG63, 143B, U2OS and SAOS2: N = 3; lncRNA-CIR high expression: n = 36, low expression: n = 18; differences among the curves were analyzed by Log-rank test; ^#^*P *< 0.05 vs hFOB1.19 cells, *P < 0.05 vs the sh-NC group, ^+^*P *< 0.05 vs the oe-NC group. The measurement data conforming to the normal distribution were expressed as mean ± standard deviation, one-way ANOVA was used for comparisons among multiple groups and Tukey’s post hoc test was used for pairwise comparisons after one-way ANOVA

The relation between lncRNA-CIR expression and the clinicopathological features of osteosarcoma patients was analyzed (Table 2), the results indicated that lncRNA-CIR was not related to the gender, age and tumor size of patients (all *P *> 0.05), while tightly associated with differentiation, disease stage and distant metastasis (all *P *< 0.05). Moreover, the follow-up data of the patients were collected to analyze the relation between lncRNA-CIR expression and prognosis of osteosarcoma patients. The results of Kaplan–Meier survival curve reflected that the high expression of lncRNA-CIR indicated a poor prognosis of osteosarcoma (*P* = 0.002; Fig. 1c).

RETRACTED

**Table 2:** Relation between lncRNA-CIR expression and clinicopathological characteristics of osteosarcoma patients

Characteristic	LncRNA-CIR		*P*
	Low expression	High expression	
All case (n = 54)	18	36	
Age (year)			0.569
< 23	8	13	
≥ 23	10	23	
Gender			0.766
Male	11	24	
Female	7	12	
Differentiation			0.012
Median/well	10	7	
Poor	8	29	
Tumor size (cm)			0.766
≥ 3	7	12	
< 3	11	24	
Disease stage			0.004
IA	3	2	
IB	3	2	
IIA	5	3	
IIB	5	5	
III	2	24	
Distant metastasis			0.008
Yes	5	25	
No	13	11	

Prognosis of patients was measured by Kaplan–Meier method and the classified variable was analyzed by Fisher’s exact test

*lncRNA-CIR* long non-coding RNA cartilage injury-related

Cox’s proportional hazards regression was employed for multivariate analysis of prognostic factors of osteosarcoma and the outcomes mirrored that (Table 3) expression of lncRNA-CIR, disease stage, distant metastasis and differentiation were the independent influence factors of prognosis of osteosarcoma patients.

**Table 3:** Measurement of independent influence factors of prognosis of osteosarcoma patients

	B	SE	Wald	df	Sig.	Exp (B)	Exp (B) 95.0% CI	
							Lower	Upper
LncRNA-CIR expression (high/low)	1.633	0.827	3.901	1	0.048	5.118	1.013	25.865
Differentiation (poor/(median + well))	1.720	0.584	8.683	1	0.003	5.583	1.779	17.524
Disease stage (III/(II + I))	2.013	0.775	6.755	1	0.009	7.489	1.641	34.184
Distant metastasis (yes/no)	3.599	1.405	6.565	1	0.010	36.557	2.330	573.479
Size (< 3 cm/≥ 3 cm)	− 2.173	1.498	2.104	1	0.147	0.114	0.006	2.145
Gender (female/male)	− 0.449	0.794	0.319	1	0.572	0.639	0.135	3.026
Age (≥ 23 years/< 23 years)	2.031	1.163	3.049	1	0.081	7.624	0.780	74.546

Cox’s proportional hazards regression was employed for multivariate analysis of prognostic factors

B: model coefficient; SE: standard error; Wald: Wald test value; df: degree of freedom; Sig: significance, *P* value; Exp (B), hazard ratio; CI: confidence interval; I: IA + IB; II, IIA + IIB

To explore the role of lncRNA‑CIR in vitro, it was either knocked down or overexpressed in MG63 and 143B cells. The knockdown and overexpression efficiency were determined by RT-qPCR. The results (Fig. 1d, e) showed that compared with the corresponding control group, the expression of lncRNA‑CIR in MG63 and 143B cells was down-regulated in the sh-CIR group, but was significantly up-regulated in the oe-CIR group (both *P *< 0.05); there was no evident difference in lncRNA-CIR expression among the control group, the oe-NC group and the sh-NC group (all *P *> 0.05).

RETRACTED

### Inhibited lncRNA-CIR restrains proliferation of MG63 and 143B cells

In order to identify the effect of lncRNA-CIR on proliferation of MG63 and 143B cells, lncRNA-CIR was reduced or overexpressed, and then colony formation, EdU and CCK-8 assays were employed to measure the proliferation of MG63 (Fig. 2a–c) and 143B cells (Fig. 3a–c). It could be found that the proliferation and colony formation ability of MG63 and 143B cells were restricted after lncRNA-CIR was inhibited, while were apparently promoted after lncRNA-CIR was overexpressed (both *P *< 0.05); no broad difference in proliferation and colony formation ability of MG63 and 143B cells could be observed among the control group, the oe-NC group and the sh-NC group (all *P *> 0.05).

**Fig. 2:** Inhibited lncRNA-CIR restrains proliferation of MG63 cells. **a** The colony formation ability of MG63 cells was determined by colony formation assay; **b** Proliferation of MG63 cells was determined by EdU assay (50 μm); **c** Viability of MG63 cells was determined by CCK-8 assay; **d** Protein expression of PCNA and Ki67 in MG63 cells was evaluated by Western blot analysis; **e** Protein bands of PCNA and Ki67 in MG63 cells; *P < 0.05 vs the sh-NC group, ^+^*P *< 0.05 vs the oe-NC group. The measurement data conforming to the normal distribution were expressed as mean ± standard deviation, one-way ANOVA was used for comparisons among multiple groups and Tukey’s post hoc test was used for pairwise comparisons after one-way ANOVA. The experiment was repeated for 3 times

**Fig. 3:** Inhibited lncRNA-CIR restrains proliferation of 143B cells. **a** The colony formation ability of 143B cells was determined by colony formation assay; **b** Proliferation of 143B cells was determined by EdU assay (50 μm); **c** Viability of 143B cells was determined by CCK-8 assay; **d** Protein expression of PCNA and Ki67 in 143B cells was evaluated by Western blot analysis; **e** Protein bands of PCNA and Ki67 in 143B cells; *P < 0.05 vs the sh-NC group, ^+^*P *< 0.05 vs the oe-NC group. The measurement data conforming to the normal distribution were expressed as mean ± standard deviation, one-way ANOVA was used for comparisons among multiple groups and Tukey’s post hoc test was used for pairwise comparisons after one-way ANOVA. The experiment was repeated for 3 times

To further confirm the function of lncRNA-CIR in osteosarcoma cell proliferation, the MG63 and 143B cells were transfected with lncRNA-CIR silenced or overexpressed plasmids, and the expression of PCNA and Ki67 in MG63 (Fig. 2d, e) and 143B cells (Fig. 3d, e) was determined by Western blot analysis. The results indicated that relative to corresponding control group, the expression levels of PCNA and Ki67 were repressed in MG63 and 143B cells in the sh-CIR group, while were elevated in Ki67 in MG63 and 143B cells in the oe-CIR group (all *P *< 0.05); there was no marked difference in protein expression of PCNA and Ki67 in MG63 and 143B cells among the control group, the oe-NC group and the sh-NC group (all *P *> 0.05).

RETRACTED

### Inhibited lncRNA-CIR promotes apoptosis of MG63 and 143B cells

LncRNA-CIR was up- or down-regulated to assess the effect of varied lncRNA-CIR on apoptosis of MG63 (Fig. 4a–c) and 143B cells (Fig. 5a–c) through TUNEL staining and Annexin V-APC/PI double staining. It came out that the apoptosis of MG63 and 143B cells was increased by reduced lncRNA-CIR, whereas suppressed by promoted lncRNA-CIR (all *P *< 0.05); there was no noticeable difference in apoptosis of MG63 and 143B cells among the control group, the oe-NC group and the sh-NC group (all *P *> 0.05).

**Fig. 4:** Inhibited lncRNA-CIR promotes apoptosis of MG63 cells. **a** Representative images of TUNEL staining of MG63 cells (50 μm); **b** Apoptosis of MG63 cells was determined by flow cytometry; **c** Comparisons of apoptosis rate of MG63 cells among the groups; **d** Protein expression of Bcl-2 and Bax in MG63 cells; **e** Protein bands of Bcl-2 and Bax in MG63 cells; *P < 0.05 vs the sh-NC group, ^+^*P *< 0.05 vs the oe-NC group. The measurement data conforming to the normal distribution were expressed as mean ± standard deviation, one-way ANOVA was used for comparisons among multiple groups and Tukey’s post hoc test was used for pairwise comparisons after one-way ANOVA. The experiment was repeated for 3 times

**Fig. 5:** Inhibited lncRNA-CIR promotes apoptosis of 143B cells. **a** Representative images of TUNEL staining of 143B cells (50 μm); **b** Apoptosis of 143B cells was determined by flow cytometry; **c** Comparisons of apoptosis rate of 143B cells among the groups; **d** Protein expression of Bcl-2 and Bax in 143B cells; **e** Protein bands of Bcl-2 and Bax in 143B cells; *P < 0.05 vs the sh-NC group, ^+^*P *< 0.05 vs the oe-NC group. The measurement data conforming to the normal distribution were expressed as mean ± standard deviation, one-way ANOVA was used for comparisons among multiple groups and Tukey’s post hoc test was used for pairwise comparisons after one-way ANOVA. The experiment was repeated for 3 times

Moreover, the expression of apoptosis-related proteins Bcl-2 and Bax in MG63 (Fig. 4d, e) and 143B cells (Fig. 5d, e) was measured by Western blot analysis, and we have found that the inhibited lncRNA-CIR suppressed the expression of Bcl-2, but up-regulated the expression of Bax in MG63 and 143B cells, and the elevated lncRNA-CIR exerted a reverse result (all *P *< 0.05); no obvious difference in protein expression of Bcl-2 and Bax could be found among the control group, the oe-NC group and the sh-NC group (all *P *> 0.05).

RETRACTED

### Inhibited lncRNA-CIR decelerates invasion and migration of MG63 and 143B cells

To explore the role of lncRNA-CIR in the invasion and migration abilities of MG63 and 143B cells, lncRNA-CIR was knocked down or overexpressed, and then the invasion and migration abilities of MG63 (Fig. 6a, b) and 143B cells (Fig. 7a, b) were evaluated by Transwell assay and scratch test, the outcomes mirrored that compared with the relative NC groups, the invasion and migration abilities of MG63 and 143B cells were reduced in the sh-CIR group, but enhanced in the oe-CIR group, separately (all *P *< 0.05); there was no obvious difference in migration abilities of MG63 and 143B cells among the control group, the oe-NC group and the sh-NC group (all *P *> 0.05).

**Fig. 6:** Inhibited lncRNA-CIR decelerates invasion and migration of MG63 cells. **a** Invasion ability of MG63 cells was evaluated by Transwell assay (25 μm); **b** Migration ability of MG63 cells was evaluated by scratch test (200 μm); **c** Protein expression of MMP2 and MMP9 in MG63 cells; **d** Protein bands of MMP2 and MMP9 in MG63 cells; *P < 0.05 vs the sh-NC group, ^+^*P *< 0.05 vs the oe-NC group. The measurement data conforming to the normal distribution were expressed as mean ± standard deviation, one-way ANOVA was used for comparisons among multiple groups and Tukey’s post hoc test was used for pairwise comparisons after one-way ANOVA. The experiment was repeated for 3 times

**Fig. 7:** Inhibited lncRNA-CIR decelerates invasion and migration of 143B cells. **a** Invasion ability of 143B cells was evaluated by Transwell assay (25 μm); **b** Migration ability of 143B cells was evaluated by scratch test (200 μm); **c** Protein expression of MMP2 and MMP9 in 143B cells; **d** Protein bands of MMP2 and MMP9 in 143B cells; *P < 0.05 vs the sh-NC group, ^+^*P *< 0.05 vs the oe-NC group. The measurement data conforming to the normal distribution were expressed as mean ± standard deviation, one-way ANOVA was used for comparisons among multiple groups and Tukey’s post hoc test was used for pairwise comparisons after one-way ANOVA. The experiment was repeated for 3 times

MMP2 and MMP9 are increased in most cancers and play vital roles in regulating invasion and metastasis [16]. Here we determined the protein expression of MMP2 and MMP9 in MG63 (Fig. 6c, d) and 143B cells (Fig. 7c, d) via Western blot analysis, the results indicated that in contrast to the NC groups, the expression of MMP2 and MMP9 in MG63 and 143B cells was declined in the sh-CIR group, but promoted in the oe-CIR group, respectively (all *P *< 0.05); there was no considerable difference in protein expression of MMP2 and MMP9 among the control group, the oe-NC group and the sh-NC group (all *P *> 0.05).

RETRACTED

### Inhibited lncRNA-CIR represses osteosarcoma tumor growth in vivo

The effect of lncRNA-CIR on osteosarcoma MG63 and 143B cells in vivo were evaluated by subcutaneous tumorigenesis in nude mice (Fig. 8a–d), the outcomes suggested that both the volume and weight of tumors were decreased in the sh-CIR group, but were increased in the oe-CIR group, which were relative to their NC groups, severally (all *P *< 0.05); no evident difference in volume and weight of tumors could be found among the control group, the oe-NC group and the sh-NC group (all *P *> 0.05).

**Fig. 8:** Inhibited lncRNA-CIR represses osteosarcoma tumor growth in vivo. **a** Morphology of transplanted tumors of nude mice that have been injected with MG63 cells; **b** Tumor volume and weight of transplanted tumors of nude mice that have been injected with MG63 cells in 6 week; **c** Morphology of transplanted tumors of nude mice that have been injected with 143B cells; **d** Tumor volume and weight of transplanted tumors of nude mice that have been injected with 143B cells in 6 week; n = 5, *P < 0.05 vs the sh-NC group, ^+^*P *< 0.05 vs the oe-NC group. The measurement data conforming to the normal distribution were expressed as mean ± standard deviation, one-way ANOVA was used for comparisons among multiple groups and Tukey’s post hoc test was used for pairwise comparisons after one-way ANOVA

RETRACTED

### Inhibited lncRNA-CIR reduces proliferation while accelerates apoptosis of osteosarcoma cells in xenografts

Immunohistochemical staining was used to assess the role of variation of lncRNA-CIR in the protein expression of Ki-67 in xenografts that separated from nude mice. We have discovered that (Fig. 9a, c) Ki-67 protein expressed in nuclei and the nuclei that stained into brownish yellow or brown indicated the Ki-67 positive expression. The Ki-67 positive cells were decreased when lncRNA-CIR was suppressed, while were increased when lncRNA-CIR was up-regulated (both *P *< 0.05); there was no apparent difference in number of Ki-67 positive cells among the control group, the sh-NC group and the oe-NC group (all *P *> 0.05). The results of Ki-67 positive cells were consistent in MG63 and 143B cells.

**Fig. 9:** Inhibited lncRNA-CIR reduces proliferation while accelerates apoptosis of osteosarcoma cells in xenografts. **a**/**c** Ki-67 expression in xenografts from nude mice that had been subcutaneously injected with MG63 and 143B cells (50 μm), and the comparisons of proliferation index among the groups; **b**/**d** Representative images of TUNEL staining in xenografts from nude mice that had been subcutaneously injected with MG63 and 143B cells (50 μm), and the comparisons of apoptotic index among the groups; n = 5, *P < 0.05 vs the sh-NC group, ^+^*P *< 0.05 vs the oe-NC group. The measurement data conforming to the normal distribution were expressed as mean ± standard deviation, one-way ANOVA was used for comparisons among multiple groups and Tukey’s post hoc test was used for pairwise comparisons after one-way ANOVA

The effect of lncRNA-CIR on apoptosis of osteosarcoma cells in vivo was evaluated by TUNEL staining in xenografts from nude mice. It came out that (Fig. 9b, d) the nuclei of apoptotic cells were stained into brownish yellow, while that of normal cells were blue. The apoptotic index of osteosarcoma cells was suppressed by overexpressed lncRNA-CIR, while was promoted by silenced lncRNA-CIR (both *P *< 0.05); no obvious difference could be observed in apoptosis index of osteosarcoma cells among the control group, the si-NC group and the oe-NC group (all *P *> 0.05). The results were consistent in MG63 and 143B cells.

## Discussion

Osteosarcoma is the commonest non-hematological malignancy of bone in children aged 15–19 years with highly aggressive and systemic metastasis, and characteristically occurs around the growth plate of long bones [17]. In recent decades, a large number of lncRNAs ranging in size from several hundred base pairs to tens of thousands base pairs have been clarified as a novel group of cancer-related non-coding RNAs (ncRNAs) in human. Among over 3000 human lncRNAs, fewer than 1% of them have been functionally identified [18]. Our research was carried out to elucidate the impacts of lncRNA-CIR on the management of osteosarcoma, and we eventually found that the inhibition of lncRNA-CIR was able to decelerate the migration, invasion and proliferation, while promote apoptosis of osteosarcoma cells, and also could suppress tumor growth in vivo.

RETRACTED

We have assessed the expression of lncRNA-CIR in osteosarcoma tissues, adjacent normal tissues, osteosarcoma cells and human normal osteoblasts. The results indicated that lncRNA-CIR was evidently up-regulated in osteosarcoma tissues and cells, which was in contrast to that in the normal tissues and osteoblasts. The elevated expression of lncRNA-CIR has been unveiled in other studies as well. For example, it has been previously confirmed that lncRNA-CIR expression was markedly augmented in OA cartilage and chondrocytes [9]. Moreover, we have measured the relation between the expression of lncRNA-CIR and characteristics of patients with osteosarcoma, and the outcomes suggested that lncRNA-CIR expression was obviously associated with differentiation, disease stage and distant metastasis, and the high expression of lncRNA-CIR was correlated with a poor prognosis of osteosarcoma patients. Similarly, a literature that studies the function of lncRNA-CIR in bladder cancer has also found that the expression of lncRNA-CIR was related with metastasis and tumor size of patients with bladder cancer, and the levels of lncRNA-CIR were associated with a poor survival [12].

In addition, the results of cellular experiments in our study unearthed that the degradation of lncRNA-CIR has the capacity to restrain proliferation, invasion and migration of osteosarcoma cells, whereas promote the cell apoptosis. Meanwhile, inhibited lncRNA-CIR also restrained tumor growth and osteosarcoma cell proliferation, whereas accelerated apoptosis of osteosarcoma cells in vivo. In view of the limited studies on role of lncRNA-CIR in human diseases, especially in malignant tumors, we referred to the study by Xiang et al., who have provided evidences that lncRNA-CIR could promote malignant phenotypes in bladder cancer cell lines. Detailedly, the study elucidated that the amplification of lncRNA-CIR could increase the viability as well as invasion of bladder cancer cells [12]. What’s more, a recent document has pointed out that the reduction of lncRNA-CIR was able to inhibit apoptosis of chondrocytes in OA [19], and Li et al. [10] have discovered that lncRNA-CIR could contribute to the degradation of chondrocyte extracellular matrix in OA. Except for cellular experiments, we have also conducted subcutaneous tumorigenesis in nude mice to observe the effect of lncRNA-CIR on osteosarcoma tumor growth in vivo, which has revealed that the suppression of lncRNA-CIR has the ability to restrain tumor growth in nude mice that had been injected with osteosarcoma cells, while the overexpressed lncRNA-CIR exerted an opposite impact. Similar to this outcome, Xiang et al. [12] have also proved that lncRNA‑CIR could increase xenograft tumor proliferation and growth in bladder cancer. All of these studies are helpful to identify the role of lncRNA-CIR in human diseases.

RETRACTED

## Conclusion

In conclusion, we have demonstrated that the repression of lncRNA-CIR could restrict the migration, invasion and proliferation, but promote apoptosis of osteosarcoma cells in vitro, and also could restrain tumor growth in vivo. This study may contribute to confirming the role of lncRNA-CIR in the progression of osteosarcoma. However, the underlying molecular mechanism of lncRNA-CIR in osteosarcoma and the correlation between lncRNA-CIR expression and tumor stem cell-like properties have not been explored in this research, which would be discussed in future work.

## Data Availability

Not applicable.

## Abbreviations

lncRNAs: long non-coding RNAs
lncRNA-CIR: lncRNA cartilage injury-related
OA: osteoarthritis
DMEM: Dulbecco’s modified Eagle medium
FBS: fetal bovine serum
P/S: penicillin–streptomycin
sh-NC: short hairpin-negative control
oe: overexpressed
RT-qPCR: reverse transcription quantitative polymerase chain reaction
NIH: National Institutes of Health
CCK-8: cell counting kit
OD: optical density
PBS: phosphate buffered saline
EdU: ethynyl-2′-deoxyuridine
APC: Annexin V-activated protein C
PI: propidium iodide
ANOVA: analysis of variance
LSD-t: least significant difference t test
ncRNAs: non-coding RNAs
